RETRACTED

# Silicon-based induced resistance in maize against fall armyworm [*Spodoptera frugiperda* (Lepidoptera: Noctuidae)]

**DOI:** 10.1371/journal.pone.0259749

**Published:** 2021-11-09

**Authors:** Inzamam Ul Haq, Aroosa Khurshid, Rehan Inayat, Kexin Zhang, Changzhong Liu, Shahbaz Ali, Ali Tan Kee Zuan, Abdulrahman Al-Hashimi, Arshad Mehmood Abbasi

**Affiliations:** 1 College of Plant Protection, Gansu Agricultural University, Lanzhou, China; 2 Department of Agricultural Engineering, Khwaja Fareed University of Engineering and Information Technology, RYK, Punjab, Pakistan; 3 Department of Land Management, Faculty of Agriculture, Universiti Putra Malaysia, Selangor, Malaysia; 4 Department of Botany and Microbiology, College of Science, King Saud University, Riyadh, Saudi Arabia; 5 Department of Environmental Sciences, COMSATS University Islamabad, Abbottabad Campus, Abbottabad, Pakistan; 6 University of Gastronomic Sciences, Pollenzo, Italy; Harran Üniversitesi: Harran Universitesi, TURKEY

## Abstract

The fall armyworm (*Spodoptera frugiperda*) is a major economic pest in the United States and has recently become a significant concern in African and Asian countries. Due to its increased resistance to current management strategies, including pesticides and transgenic corn, alternative management techniques have become more necessary. Currently, silicon (Si) is being used in many pest control systems due to its ability to increase plant resistance to biotic and abiotic factors and promote plant growth. The current experiments were carried out at the College of Plant Protection, Gansu Agricultural University, Lanzhou, China, to test the effect of Si on lifetable parameters and lipase activity of fall armyworm and vegetative and physiological parameters of maize plants. Two sources of Si (silicon dioxide: SiO_2_ and potassium silicate: K_2_SiO_3_) were applied on maize plants with two application methods (foliar application and soil drenching). The experiment results revealed that foliar applications of SiO_2_ and K_2_SiO_3_ significantly (P≤0.05) increased mortality percentage and developmental period and decreased larval and pupal biomass of fall armyworm. Similarly, both Si sources significantly (P≤0.05) reduced lipase activity of larvae, and fecundity of adults, whereas prolonged longevity of adults. Among plant parameters, a significant increase in fresh and dry weight of shoot, stem length, chlorophyll content, and antioxidant activity was observed with foliar applications of Si. Root fresh and dry weight was significantly (P ≤ 0.05) higher in plants treated with soil drenching of SiO_2_ and K_2_SiO_3_. Moreover, SiO_2_ performed better for all parameters as compared to K_2_SiO_3_ and control treatment. The study conclusively demonstrated a significant negative effect on various biological parameters of fall armyworm when plants were treated with Si, so it can be a promising strategy to control this pest.

RETRACTED

## Introduction

Maize (*Zea mays* L.) is an important agricultural crop that is used in a variety of foods, industrial and medicinal products. Due to its productivity and adaptability, it is the third most cultivated crop worldwide after wheat and rice. Several insect pests constantly threaten the production of maize crop. The fall armyworm [*Spodoptera frugiperda* (Smith) (Lepidoptera: Noctuidae)] is an important pest of maize crop. Besides maize, it also damages various other essential crops, including wheat, cotton, sugarcane, and rice [1]. Depending on environmental factors, fall armyworm goes through 6 to 7 instars before the pupal stage. The entire life cycle of the pest is temperature-dependent, which can be completed in four weeks under favorable conditions. Where host plant is available, this species can produce multiple generations throughout the year. Relatively shorter life span and multivoltine ability allow fall armyworm to infest crop fields in a short time. While fall armyworm is native to North America, where it is a severe crop pest, it has recently been reported in South Africa. Due to insufficient pest control strategies and lack of natural enemies, it destroyed entire maize fields [2] and spread over the whole continent within a short time [3]. In 2018 fall armyworm was first time reported in India [4] and Myanmar [5], and in early 2019 it was confirmed in China and other neighboring countries [3].

Usually, pesticides are used to control fall armyworm. Mainly, pesticides are applied in the later stages of the crop when the insect population is high in the fields. Therefore, these pesticides are not so effective and have side effects on human health and the environment. Damage caused by fall armyworm has urged the introduction of some alternative control methods such as resistant plants [6], biological control [7], and resistance elicitors [8]. Extracts of organic origin and essential oils obtained from plants are alternative control methods, which play a vital role in pest control. Essential oils obtained from plants are effective on insects, especially on nutrition, mating, egg-laying, and hatching [9]. It is known that dusts, like diatomaceous earth (DE), have insecticidal or repellant activity and effectively control most insects commonly found in storage products [10]. Ciniviz and Mutlu [11] treated maize grains with two local diatomaceous earth (Aydın and Ankara) and Silicosec to investigate their effect against *S*. *zeamais* adults. Induced resistance in plants can cause mechanical barriers or can cause changes in biochemical responses of plants insect attack by increased synthesis of proteins which can act as poisons and can cause changes in insect metabolism [12]. It is reported that plant resistance can be induced by applying silicon (Si) which can be an alternative for integrated management of pests. Si is the second most abundant element after Oxygen in Earth’s crust which comprises its 28% [13]. For the plant’s growth, it is not considered an essential element, but it is reported in the literature that it affects plant growth and development positively [14]. Moreover, by International Plant Nutrition Institute, Si is listed as a beneficial substance [15].

RETRACTED

Si application results in its deposition in epidermal cells of plants, which increases mechanical defense [16]. Two primary mechanisms of Si-based plant defenses involve strengthening physical or mechanical barriers and inducing plant defense mechanisms via biochemical or molecular reactions. Similarly, Si-mediated mechanisms act in plants below and above ground, as Si induces the accumulation of lignin in the roots of sugarcane [17] and oilseed rape [18], increasing toughness and, eventually, the resistance to insects [19]. Despite the differences in Si accumulation among plant species, they display similar Si defense mechanisms against insects. In addition to direct and indirect effects on plant defenses, Si can also affect the growth of immature insects and the rate of population increase [35]. It is also reported that Si application can mitigate the harmful effects of other factors such as heavy metal toxicity [20], salinity [14], and drought [21] in plants.

Keeping in view the expenses for control of fall armyworm, the use of resistance inducers is a promising alternative since the induction of resistance can keep the population of pests below the economic injury level, with minimum side effects on the environment and compatible with insect control methods. This work aims to evaluate whether foliar and drenching applications of Si increase maize resistance against fall armyworm and promote the growth and development of plants. It is expected that the results of this work can provide insights into the role of Si on maize resistance to consider its use as an alternative in integrated pest management in maize.

## Materials and methods

### Experimental site and treatments

Certified maize seeds of Nonghua-816 were planted in 25cm diameter pots using standard Pro-mix potting soil at the College of Plant Protection, Gansu Agricultural University, Lanzhou, China (36.0915° N, 103.7006° E). The seeds were purchased from the local market. Pots were kept in a temperature-controlled environment and watered daily to maintain moisture levels. The experiment was conducted in a completely randomized design (CRD) under a factorial arrangement with three replications. Treatments consisted of silicon compounds Silicon dioxide (SiO_2_) and Potassium silicate (K_2_SiO_3_) were applied by two different application methods (Foliar application and soil drenching). However, only water was applied as foliar application and soil drenching to plants under control treatment. Foliar treatments were applied using a 1 L spray bottle with the base of the plants covered with plastic to prevent soil absorption, while drenches were applied directly to the soil near the bottom of the plant. The first silicon treatment was applied to the plants after 15 days of seedling emergence, while the following silicon treatments were applied at ten days intervals. For each silicon treatment, an equal application volume of 30 ml/pot was used. Plant samples were collected and transferred to Petri dishes to assess the impact of Si on fall armyworm and check plants’ vegetative characteristics.

RETRACTED

### Insect culture

Fall armyworm eggs received from a laboratory colony were kept for hatching in the insect rearing room. Newly-emerged larvae were provided with an artificial diet to maintain the colony. Artificial diet composition is as follows: Component (a) Maize powder (150 g), Soybean powder (87g), Yeast powder (30 g), Casein (15 g), Sucrose (10 g), and distilled water 300 ml, Component (b) Agar powder (15 g) and Distilled water 350 ml, Component (c) Ascorbic acid (1.5 g), Cholesterol (0.48 g), Inositol (0.17 g), Sorbic acid (1 g), Methyl parahydrobenzoate (1.40 g), Multi-Vitamin B (0.5 g), Wesson’s salt (0.25 g) Distilled water 35 ml, Component (d) Colza oil 2 ml. Artificial diet preparation: Component (a) and Component (b) were sterilized separately at 121°C for 20 minutes, then Component (b) was added into Component A and cooled at 60°C. All the components of (c) were added into a beaker, dissolved in warm water, and then added to (a) and (b) mixture, and Component (d) was mixed.

### Data collection for fall armyworm

The fall armyworm larvae were individually placed in Petri dishes (9 cm diameter) and fed with discs of leaves from plants treated with silicon applications. In the laboratory, leaves were washed in water and replaced daily during the larval period. The Fall armyworm biological parameters evaluated were lipase activity, larval duration, survival, and biomass after 15 days of emergence; pupal duration, survival, and biomass after 24 h of formation; longevity and total fecundity of adults. The measuring method of lipase was according to Reagent Kit Sino Best Biological Technology Co., Ltd. Shanghai, China. Larval and pupal biomass was measured on a precision scale (AR224CN, Ohaus Corporation, Shanghai, China). Only values for those caterpillars that reached the pupal stage were considered in the calculation of larval duration and biomass, and similarly, duration and biomass of the pupal stage were determined only for those pupae from which adults emerged. After adult emergence, single males and females from each treatment group were paired. Each pair was isolated in cages (10 cm height × 10 cm diameter), according to the emergence date, with a total of five pairs/treatment. Cages were provided with maize plants sown in pots as an oviposition site and fed with an aqueous honey solution [15% (w:v)]. Freshly laid eggs were collected from the cages and put in clean Petri dishes (diameter, 9 cm). The numbers of eggs laid overnight were counted with the aid of a microscope. This repeated daily until females died.

RETRACTED

### Data collection for maize

The following vegetative characteristics were analyzed in maize plants 40 days after emergence: stem length, fresh and dry weight of plant shoot and root matter, chlorophyll content (using a portable chlorophyll meter), and antioxidant enzymes activity. The antioxidant activity, i.e., peroxidase (POD), superoxide dismutase (SOD), and catalase (CAT), were recorded using a spectrophotometer. The samples of maize leaves were first ground into powder in liquid nitrogen. A phosphate buffer of 7.8 pH and 0.05 M was used for maize homogenates. Homogenized and filtered solution samples were correctly centrifuged for at least 10 minutes at 12000×g at 4°C, and the mixtures were used for further examination of antioxidants analysis. The enzymatic activities of SOD and POD were documented according to the procedure mentioned by Zhang [22]. The activity of catalase (CAT) was recorded following the procedure mentioned by Aebi [23]. Briefly, H_2_O_2_ solution having a volume of 100 μl (300mM), 100 μl enzyme extract, 2.8 mL phosphate buffer @ 50mM were added in 3mL of assay mix. The observations of the CAT activity were taken at the absorbance at 240 nm wavelength. All the reagents used were of analytical quality purchased and provided by the College of Plant Protection, Gansu Agricultural University, Lanzhou, China.

### Statistical analysis

The data regarding all parameters of fall armyworm and maize were subjected to analysis of variance (factorial design up to two-way interaction) to test the effect of Si application methods and Si sources. Treatment means with significant differences were separated using the LSD test at p ≤ 0.05. All statistical analyses were carried out using SPSS statistics software (IBM, SPSS Version 19, United States). All the graphs were made by use GraphPad Prism version 7.00.

RETRACTED

## Results

### Larva survival percentage

Foliar application of SiO_2_ resulted in a significantly (P ≤ 0.05) lower survival percentage (57.00 ± 2.00%) compared to soil drenching of SiO_2_ and foliar application and soil drenching of K_2_SiO_3_ (Fig 1a). Moreover, a lower survival percentage (73.44 ± 6.19%) was observed for foliar application than drenching (77.33 ± 5.96%). Among Si sources, plants treated with SiO_2_ had a lower survival percentage of fall armyworm larva (60.00 ± 3.58%) compared to K_2_SiO_3_ (70.83 ± 3.31%) and control (95.33 ± 3.27%) (Table 1).

**Fig 1:** Effect of silicon sources and silicon application methods on (a) larva survival percentage, (b) larva duration (days), (c) larva biomass (mg), and lipase activity (U/mg protein) of fall armyworm. Means with different lower-case letters are significantly different; LSD test at p ≤ 0.05. Vertical bars indicate SD.

**Table 1:** Effect of silicon sources and silicon application methods on larva survival %, larva duration (days), biomass(mg), and lipase activity (U/mg protein) of fall armyworm feeding on maize plants.

	Larva survival (%)	Larva duration (days)	Larva biomass (mg)	Lipase activity (U/mg protein)
**Sources (S)**				
SiO_2_	60.00 ± 3.58 c	21.833 ± 1.47 a	215.33 ± 14.86 c	1.7696 ± 0.175 b
K_2_SiO_3_	70.833 ± 3.31 b	19.167 ± 1.72 b	255.50 ± 10.46 b	1.8183 ± 0.167 b
Control	95.33 ± 3.27 a	15.50 ± 0.54 c	294.67 ± 8.82 a	2.2672 ± 0.134 a
**Application methods (M)**				
Foliar	73.44 ± 6.19 b	19.778 ± 1.48 a	247.78 ± 24.76 b	1.8664 ± 0.319 b
Drenching	77.33 ± 5.96 a	17.889 ± 1.73 b	262.56 ± 19.75 a	2.0370 ± 0.190 a
F value (S)	441.26	140	243.96	187.78
F value (M)	15.27	37.05	25.39	54.47
F value (S×M)	3.83	6.67	7.13	17.54

Means within a column followed by different lower-case letters are significantly different at P ≤ 0.05 (LSD test)

### Larva duration (days)

Significantly (P ≤ 0.05) prolonged larval duration (23.00 ± 1.00 days) of fall armyworm was observed on the plants treated with foliar applications of SiO_2_ and compared to those plants treated with foliar applications and soil drenching K_2_SiO_3_(Fig 1b). Moreover, larval duration was also influenced significantly (P ≤ 0.05) by plants treated with foliar application of Si (19.778 ± 1.47 days) compared to soil drenching (17.889 ± 1.72 days). Among Si sources, SiO_2_ caused a significant (P ≤ 0.05) increase in larval duration (17.889 ± 1.72 days) compared to K_2_SiO_3_ (17.889 ± 1.72 days) (Table 1).

RETRACTED

### Larva biomass (mg)

The larva biomass of fall armyworm was significantly (P ≤ 0.05) affected by all treatments. The lowest biomass (202 ± 2.65 mg) was recorded in larvae fed on plants treated with foliar application of SiO_2_ (Fig 1c). Among application methods, lower biomass (247.78 ± 24.77 mg) was recorded in the foliar application than soil drenching (262.56 ± 19.76 mg). Similarly, lower biomass (215.33 ± 14.87 mg) of fall armyworm larvae was recorded on plants treated with SiO_2_ compared to K_2_SiO_3_ (255.50 ± 10.46 mg) and control (294.67 ± 8.82 mg) (Table 1).

### Lipase activity (U/mg protein)

Results of the current study indicated that the lipase activity of fall armyworm larvae was negatively affected by Si application. Foliar application of SiO_2_ (1.6316 ± 0.104 U/mg protein) as well as of K_2_SiO_3_ (1.6890 ± 0.113 U/mg protein) significantly (P ≤ 0.05) affected lipase activity compared to soil drenching (Fig 1d). Among Si sources, lipase activity was significantly (P ≤ 0.05) more affected by SiO_2_ (1.7696 ± 0.175 U/mg protein) compared to K_2_SiO_3_ (1.8183 ± 0.167 U/mg protein) and control (2.2672 ± 0.134 U/mg protein). Significantly lower values of lipase activity were recorded in insects fed on plant leaves treated with a foliar application (1.8664 ± 0.319 U/mg protein) compared to soil drenching (2.037 ± 0.190 U/mg protein) (Table 1).

### Pupa survival percentage

Pupa survival percentage of fall armyworm was significantly (P ≤ 0.05) influenced by the plants treated with foliar application of SiO_2_ (89.67 ± 0.58 (Fig 2a). Among application methods, a significantly (P ≤ 0.05) lower survival percentage was observed in foliar applications (93.778 ± 4.76%) compared to soil drenching (95.34 ± 3.54%). A lower survival percentage of fall armyworm pupa was observed in SiO_2_ (91.17 ± 1.72%) treated plants compared to K_2_SiO_3_ (92.50 ± 1.04%) and control (100 ± 0.00%) (Table 2).

**Fig 2:** Effect of silicon sources and silicon application methods on (a) pupal survival percentage, (b) pupa duration (days), and (c) pupa biomass (mg) of fall armyworm. Bars with different lower-case letters are significantly different; LSD test at p ≤ 0.05. Vertical bars indicate SD.

**Table 2:** Effect of silicon sources and silicon application methods on pupa survival percentage, pupa duration (days), and pupa biomass(mg) of fall armyworm feeding on maize plants.

	Pupa survival (%)	Pupa duration (days)	Pupa biomass (mg)
**Sources (S)**			
SiO_2_	91.17 ± 1.72 c	10.162 ± 0.58 a	171.16 ± 9.41 c
K_2_SiO_3_	92.50 ± 1.05 b	9.56 ± 0.24 b	181.17 ± 9.78 b
Control	100 ± 00 a	9.04 ± 0.09 c	197.67 ± 1.63 a
**Application methods (M)**			
Foliar	95.333 ± 3.54 a	9.826 ± 0.72 a	177.56 ± 15.78 b
Drenching	93.778 ± 4.76 b	9.347 ± 0.28 b	189.11 ± 7.85 a
F value (S)	612.25	90.75	467.17 ±
F value (M)	49.00	49.54	261.26
F value (S×M)	15.25	18.51	65.39

Means within a column followed by different lower-case letters are significantly different at P ≤ 0.05 (LSD test).

RETRACTED

### Pupa duration (days)

Significantly (P ≤ 0.05) longer pupa duration of fall armyworm was observed in the foliar application of SiO_2_ (10.67 ± 0.29 days (Fig 2b). Soil drenching of SiO_2_ (9.65 ± 0.04 days) and foliar application of K_2_SiO_3_ (9.77 ± 0.02 days) were significantly similar in impact on pupa duration. Overall, a significantly (P ≤ 0.05) prolonged pupa duration was observed in the foliar application (9.83 ± 0.72 days) compared to soil drenching (9.35 ± 0.28 days). Moreover, a significantly (P ≤ 0.05) extended pupa duration was observed on the plants treated with SiO_2_ (10.16 ± 0.58 days) compared to K_2_SiO_3_ (9.56 ± 0.24 days) and control (9.04 ± 0.09 days) (Table 2).

### Pupa biomass (mg)

Foliar applications of SiO_2_ significantly (P ≤ 0.05) influenced the pupa biomass (162.67 ± 2.08 mg) compared to soil drenching and foliar application and soil drenching of K_2_SiO_3_ (Fig 2c). Among application methods, significantly (P ≤ 0.05) lower pupa biomass was recorded in the foliar application (177.56 ± 15.77 mg) compared to soil drenching (189.11 ± 7.85 mg) of Si. Moreover, significantly (P ≤ 0.05) lower biomass was recorded in plants treated with SiO_2_ (171.17 ± 9.41 mg) compared to K_2_SiO_3_ (181.16 ± 9.79 mg) and control (197.67 ± 1.63 mg) (Table 2).

### Fecundity

Maize plants treated with foliar applications of SiO_2_ significantly (P ≤ 0.05) influenced the fecundity (130.00 ± 2.65 eggs) of fall armyworm better compared to soil drenching and foliar applications and soil drenching of K_2_SiO_3_ (Fig 3a). A significantly lower fecundity (154.33 ± 28.27 eggs) was observed in treatments receiving foliar applications than soil drenching (174.22 ± 13.10 eggs). Among Si sources, a significantly (P ≤ 0.05) lower fecundity was recorded in SiO_2_ (146.67 ± 18.36 eggs) compared to K_2_SiO_3_ (154.83 ± 14.52 eggs) and control (191.33 ± 2.25 eggs) (Table 3).

**Fig 3:** Effect of Si sources and application methods on (a) adult fecundity (n) and (b) adult longevity (days) of fall armyworm. Bars with different lower-case letters are significantly different; LSD test at p ≤ 0.05. Vertical bars indicate SD.

**Table 3:** Effect of Si sources and Si application methods on adult fecundity (n) and adult longevity (days) of fall armyworm feeding on maize plants.

	Longevity (days)	Fecundity (n)
**Sources (S)**		
SiO_2_	9.667 ± 1.21 c	146.67 ± 18.36 c
K_2_SiO_3_	10.883 ± 0.98 b	154.83 ± 14.52 b
Control	12.500 ± 0.54 a	191.33 ± 2.25 a
**Application methods (M)**		
Foliar	10.333 ± 1.65 b	154.33 ± 28.27 b
Drenching	11.667 ± 1.01 a	174.22 ± 13.10 a
F value (S)	40.56	662.61
F value (M)	26.67	347.52
F value (S×M)	3.89	90.47

Means within a column followed by different lower-case letters are significantly different at P ≤ 0.05 (LSD test).

RETRACTED

### Longevity

A significantly (P ≤ 0.05) shorter adult longevity (8.67 ± 0.58 days) of fall armyworm was recorded in the insects fed on plants receiving the foliar application of SiO_2_. There was no significant difference found between soil drenching of SiO_2_ (10.00 ± 0.00 days) and foliar application of K2SiO_3_ (10.67 ± 0.57 days) (Fig 3b). Adult longevity was significantly shorter in the foliar application (10.34 ± 1.65 days) of Si than soil drenching (11.67 ± 1.00 days). Among Si sources, SiO_2_ resulted in significantly (P ≤ 0.05) shorter longevity (9.67 ± 1.21 days) of the adult compared to K_2_SiO_3_ (10.83 ± 0.98 days) and control (12.50 ± 0.54 days) (Table 3).

### Effect of Si on fresh and dry biomass of maize

(Fig 4) shows the result of analysis of variance for the effect of SiO_2_ and K_2_SiO_3_ on fresh and dry biomass of shoot and root. SiO_2_ has a significant impact (p ≤ 0.05) on fresh biomass (25.70 ± 0.26 g) and dry biomass (3.64 ± 0.05 g) of the shoot when applied as a foliar application. While both SiO_2_ and K_2_SiO_3_, when used as soil drenching, had a significantly similar effect on fresh biomass (23.23 ± 0.11 g), (23.12 ± 0.04 g) and dry biomass (3.38 ± 0.26 g), (3.31 ± 0.25 g) of shoot respectively. Fresh biomass (13.91 ± 0.02 g) and dry biomass (2.19 ± 0.025 g) of root were significantly (p ≤ 0.05) affected by SiO_2_ when applied as soil drenching. Among application methods, shoot fresh biomass (23.78 ± 2.13 g) and dry biomass (3.32 ± 0.39 g) of plants treated with foliar applications of SiO_2_ and K_2_SiO_3_ were significantly (p ≤ 0.05) more compared to shoot fresh biomass (22.46 ± 1.15 g) and dry biomass (3.15 ± 0.30 g) of plants treated with soil drenching of Si. While soil drenching significantly (p ≤ 0.05) resulted in an increase in fresh biomass (12.987 ± 1.01 g) and dry biomass (1.99 ± 0.26 g) of the roots compared to biomasses (12.29 ± 0.48 g), (1.82 ± 0.14 g) in foliar applications of SiO_2_ and K_2_SiO_3_. Moreover, among Si sources, significantly (p ≤ 0.05) more fresh and dry biomass of the shoot (24.67 ± 1.36 g), (3.51 ± 0.14 g), as well as root (13.33 ± 0.65 g), (2.07 ± 0.13 g), were recorded in those plants which were treated with SiO_2_ compared to K_2_SiO_3_ and control (Table 4).

**Fig 4:** Effect of Si sources and Si application methods on (a) shoot fresh weight (g), (b) shoot dry weight (g), (c) root fresh weight (g), and (d) root dry weight (g) of maize. Bars with different lower-case letters are significantly different; LSD test at p ≤ 0.05. Vertical bars indicate SD.

RETRACTED

**Table 4:** Effect of Si sources and Si application methods on shoot fresh weight (g) shoot dry weight (g), root fresh weight (g), and root dry weight (g) of maize plants.

	Shoot fresh weight (g)	Shoot dry weight (g)	Root fresh weight (g)	Root dry weight (g)
**Sources (S)**				
SiO_2_	24.467 ± 1.36 a	3.5133 ± 0.14 a	13.330 ± 0.65 a	2.0733 ± 0.13 a
K_2_SiO_3_	23.872 ± 0.83 b	3.4200 ± 0.12 b	12.905 ± 0.51 b	1.9950 ± 0.16 b
Control	21.025 ± 0.58 c	2.7833 ± 0.07 c	11.693 ± 0.17 c	1.6483 ± 0.03 c
**Application methods (M)**				
Foliar	23.782 ± 2.13 a	3.3267 ± 0.39 a	12.299 ± 0.48 b	1.8189 ± 0.14 b
Drenching	22.460 ± 1.15 b	3.1511 ± 0.30 b	12.987 ± 1.01 a	1.9922 ± 0.26 a
F value (S)	123.51	480.15	329.95	377.90
F value (M)	47.86	70.32	162.30	166.46
F value (S×M)	13.81	7.92	46.21	41.18

Means within a column followed by different lower-case letters are significantly different at P ≤ 0.05 (LSD test).

### Effect of Si on stem length (cm) and chlorophyll index (SPAD value)

Stem length and chlorophyll index of maize plants were significantly (p ≤ 0.05) influenced by different Si sources and application methods. Significantly (p ≤ 0.05), more chlorophyll content (38.52 ± 0.26) and longer stem length (51.39 ± 0.62 cm) was recorded in plants that were treated with foliar application of SiO_2_ (Fig 5). Stem length was significantly (p ≤ 0.05) similar in plants treated with soil drenching of SiO_2_ (46.07 ± 0.09 cm) of K_2_SiO_3_ (45.67 ± 0.29 cm). Foliar application of both Si sources resulted in significantly increased stem length (47.05 ± 4.27 cm) and chlorophyll content (34.52 ± 4.88) compared to soil drenching. Similarly, plants treated with SiO_2_ were significantly (p ≤ 0.05) taller (47.05 ± 4.27 cm) and with more chlorophyll content (47.05 ± 4.27 cm) compared with K_2_SiO_3_ and control (Table 5).

**Fig 5:** Effect of Si sources and Si application methods on (a) stem length (cm) and chlorophyll content (SPAD value) of maize. Bars with different lower-case letters are significantly different; LSD test at p ≤ 0.05. Vertical bars indicate SD.

**Table 5:** Effect of silicon sources and silicon application methods on stem length (cm) and chlorophyll index (SPAD value) of maize plants.

	Stem length (cm)	Chlorophyll index (SPAD value)
**Sources (S)**		
SiO_2_	48.730 ± 2.95 a	34.763 ± 4.12 a
K_2_SiO_3_	46.790 ± 1.24 b	33.603 ± 3.68 b
Control	41.670 ± 1.05 c	28.057 ± 0.28 c
**Application methods (M)**		
Foliar	47.048 ± 4.27 a	34.517 ± 4.89 a
Drenching	44.412 ± 2.20 b	29.766 ± 1.35 b
F value (S)	147.23	1697.32 ±
F value (M)	57.66	2236.49
F value (S×M)	17.56	561.27

Means within a column followed by different lower-case letters are significantly different at P ≤ 0.05 (LSD test).

RETRACTED

### Effect of Si on antioxidant enzymes activity of maize plants

Results of this study indicated that superoxide dismutase (SOD), (peroxidase) POD, and catalase (CAT) activities significantly (p ≤ 0.05) increased in all Si treatments compared to control. Foliar application of SiO_2_ resulted in significantly (p ≤ 0.05) higher values of SOD (0.150 ± 0.007 g^-1^ FW), POD (0.435 ± 0.02 g^-1^ FW), and CAT (0.209 ± 0.04 g^-1^ FW) (Fig 6). SOD activity was significantly (p ≤ 0.05) similar in soil drenching of SiO_2_ (0.100 ± 0.02 g^-1^ FW) as well as foliar applications (0.120 ± 0.02 g^-1^ FW) and soil drenching (0.103 ± 0.08 g^-1^ FW) of K_2_SiO_3_. POD activity was significantly (p ≤ 0.05) similar in soil drenching of both Si sources. Among Si application methods, significantly (p ≤ 0.05) higher values of SOD (0.108 ± 0.04 g^-1^ FW), POD (0.279 ± 0.17 g^-1^ FW), and CAT (0.157 ± 0.07 g^-1^ FW) were recorded in those plants which receive foliar applications of both Si sources compared to soil drenching. Moreover, significantly (p ≤ 0.05) higher values of POD (0.313 ± 0.14 g^-1^ FW) were recorded in the plants treated with SiO_2_ compared to K_2_SiO_3_ and control, while SOD and CAT activities were significantly similar in both Si sources (Table 6).

**Fig 6:** Effect of Si sources and Si application methods on antioxidant enzymes activity of maize. Bars with different lower-case letters are significantly different; LSD test at p ≤ 0.05. Vertical bars indicate SD.

**Table 6:** Effect of silicon sources and silicon application methods on antioxidant enzymes activity (SOD, POD, and CAT) of maize plants.

	SOD (g^-1^ FW)	POD (g^-1^ FW)	CAT (g^-1^ FW)
**Sources (S)**			
SiO_2_	0.1250 ± 0.03 a	0.3129 ± 0.14 a	0.1831 ± 0.04 a
K_2_SiO_3_	0.1118 ± 0.02 a	0.2581 ± 0.09 b	0.1653 ± 0.03 a
Control	0.0553 ± 0.005 b	0.0646 ± 0.007 c	0.0748 ± 0.008 b
**Application methods (M)**			
Foliar	0.1082 ± 0.04 a	0.2788 ± 0.17 a	0.1570 ± 0.07 a
Drenching	0.0866 ± 0.03 b	0.1449 ± 0.06 b	0.1252 ± 0.04 b
F value (S)	55.30	494.10	79.65
F value (M)	14.21	389.99	17.91
F value (S×M)	6.64	118.38	7.92

Means within a column followed by different lower-case letters are significantly different at P ≤ 0.05 (LSD test).

## Discussion

In the current study, foliar applications and soil drenching of Si significantly affected the growth parameters of fall armyworm. Application of both Si sources caused a decrease in survival percentage, extended larval and pupal duration, and reduced biomass and lipase activity of larvae compared to untreated control. Sublethal effects of Si on fall armyworm adult and reproductive parameters were also detected.

RETRACTED

Higher concentrations of Si in leaves can cause mechanical protection and biochemical changes in plants which can increase the defense levels of plants and affect the development of fall armyworm [24]. Brunings et al. [25] reported differential expression of 221 genes in Si treated rice, 28 of which involved plant defense. Hence, it’s evidence that Si also acts as a plant resistance elicitor. Insect development can be affected negatively by Si application. These effects can be direct by affected growth or indirect by delay in establishing insects on plants, increasing exposure of insects to adverse abiotic factors, and natural enemies [24]. The harmful effects of plants treated with Si on the development of fall armyworm may have resulted from polymerization and accumulation of silicate compounds in the cell walls of plants that increased the rigidity and decreased digestibility of leaf tissues which resulted in reduced growth rates of larvae [16]. Si application can enhance the synthesis of secondary defense compounds that can affect fall armyworm on plants [26]. Si is translocated within the plant in the form of mono silicic acid, and—when concentrated over a critical level—it polymerizes as opaline phytoliths mainly in the leaf epidermal cells, which comprise the bulk of a plant’s Si content [27].

Results of this study are in line with the findings of Mondego et al. [28], who reported that when fall armyworm larvae fed with Si treated plants, their viability percentage was decreased (64%) as compared to control (92%). He further stated that K_2_SiO_3_ negatively affected the viability of fall armyworm when applied alone and with another growth inhibitor. The larval period extension observed in the treatment of K_2_SiO_3_ may be related to a food substrate nutritional inadequacy that probably extended the larval period. This type of response is desirable in integrated pest management programs since the increase of the larval stage may favor the action of natural enemies. Therefore, the caterpillars will be exposed for a longer time. In addition, they will complete fewer generations per corn phenological cycle. Similarly, Hou and Han [29] reported that compared with the control, the Si accumulation in rice plants treated with calcium silicate was more prominent. The high Si content was directly related to the prolonged larval development and penetration time of *Chilo suppressalis*, as well as the reduction of borer infestation, weight gain, and stem damage. In general, these studies indicated that Si-induced antibiotic activity could antagonize herbivorous insects with different feeding habits. Moreover, he reported that prolonged larval (20.18 days) and pupal duration (10.46 days) was recorded in the treatments consisting of potassium silicate as compared to untreated control where the shorter period of larvae (17.40 days) and pupae were recorded. Massey and Hartley [16] observed a decrease in larval weight of *Spodoptera exempta* fed on Si-treated plants, which decreased the efficacy of larvae in converting ingested food into live biomass. Mondego et al. [28] reported that maize leaves treated with K_2_SiO_3_ had the lowest weight gain for male and female pupae of fall armyworm, significantly different from the control. In this study, the effectiveness of spraying SiO_2_ and K_2_SiO_3_ on the leaf surface may be due to the anti-nutrition effect observed in the larval stage of fall armyworm, which directly affects the weight of pupae. A lower weight of pupae may induce changes in the fecundity of insects which results in smaller moths and infertile eggs [26]. It is a desirable factor in IPM because it may reduce the pest population and damage to crops, reducing the cost of pesticide application.

RETRACTED

The midgut epithelium of insects plays a vital role in the digestion and converting food to nutrients by digestive enzymes [30]. There are many Endogenic enzyme inhibitors like protease inhibitors that bind to endopeptidases and exopeptidases in insects and efficiently inhibit growth [31], similarly some a-amylase inhibitors [32], and trypsin-modulating oostatic factor (TMOF) that efficiently inhibit translation of trypsin mRNA in the gut of *Heliothis virescens* larvae [33]. Si could also destroy the structure of the epithelium of the midgut, mainly by the detachment of epithelial cells from the basement membrane as detected in larvae of *Tuta absoluta* fed with tomato leaves treated with Si [34]. This negatively affects the nutrient absorption, enzyme activity, and growth rate of insects [35]. The current study results clearly show that the lipase activity of fall armyworm was negatively affected by silicon applications.

Abbasi et al. [36] observed lower fecundity of whitefly adults derived from nymphs fed on cotton plants treated with Si. He reported foliar Si applications oviposited a smaller number of eggs (75.05 eggs) than drenching silicon applications (87.08 eggs). Among Si sources, plants treated with SiO_2_ had a significantly lower number of oviposited eggs (77.03) than K_2_SiO_3_ treated cotton plants (85.10). Alvarenga et al. [37] indicated that treatment with Si and gibberellic acid affected adult phase parameters of fall armyworm. When females were derived from larvae fed with plants treated with these substances, their fecundity was adversely affected. Insect fecundity is one of the biological parameters most affected by Si. Silva et al. [38] reported that male-female pairs of fall armyworm derived from larvae fed on cotton leaves treated with Si produced fewer eggs per female. At the same time, He et al. [39] demonstrated that feeding with rice plants treated with Si solution significantly reduced the fecundity of *Nilaparvata lugens* (Stal). This deleterious effect on oviposition may be due to the accumulation of Si in plants, which can activate and increase the production of defense metabolites [40]. Additional studies (mainly of aphids) have also suggested that Si reduces insect fecundity [41]. Results of the current study are well supported by the findings of Mondego et al. [28], who reported that treatments consisted of K_2_SiO_3_ resulted in a prolonged developmental period (12.26) of fall armyworm adults compared to control. Similarly, Abbasi et al. [36] observed the extended longevity of *B*. *tabaci* on plants treated with foliar applications of SiO_2_ compared to soil drenching and untreated control.

RETRACTED

Results of this study showed that Si applications not only affected the performance of insects but also positively affected the vegetative and physiological parameters of the maize plant. Positive effects of Si applications were observed on stem length, fresh & dry weights of shoots and roots, chlorophyll content, and antioxidant enzymes activity of maize plants. Results of the current study are in line with previous findings of Francis and Sorrell [42], who reported that with applications of Si and gibberellic acid, an increase in elongation of internodes was observed. Similar results are reported by Rohanipoor et al. [43], who observed significantly increased stem length with the application of Si. Furthermore, he reported that Si significantly (p<0.01) affected the fresh and dry weight of shoot, dry weight of root, and significantly (p<0.05) affected the fresh weight of root. Maize plants treated with higher concentrations of Si resulted in an increase in fresh and dry weight of shoot and root compared to those treated with lower concentrations of Si and control. It is reported in many studies that Si application has a positive effect on the growth development and yield of plants. Dresler et al. [44] observed an increase in the dry weight of barley when treated with Si compared to those plants receiving no Si application. Barker and Pilbeam [45] reported that Si treatments resulted in an increase in mass and volume of the roots, which increased adsorbing surface of roots. Moreover, he observed fresh weight and dry weight of both shoot and root in plants with the application of Si were increased.

RETRACTED

Results of the current study are well supported by Al-aghabary [46] in *Lycopersicon esculentum*, Amirossadat [47] in *Cucumis sativus*, and Moussa [48] in *Zea mays*. They reported that applications of Si significantly increased chlorophyll content. Liang et al. [49] said that Si application increased H^+^-ATPase activity, minimized damage to the chloroplast, and thus increased chlorophyll and photosynthetic activity of leaves.

The defense mechanism of antioxidant stress is critical for eliminating reactive oxygen species by various enzymatic and non-enzymatic antioxidant molecules [50]. If this system does not work correctly, plants can be affected by reactive oxygen species damage [51]. The results of the current study showed that antioxidant enzymatic activity was increased in maize with Si application. Liang et al. [52] reported that superoxide dismutase, peroxidase, and catalase activity were significantly increased in barley leaves with Si application. Tale Ahmad [53] reported that CAT activity was significantly increased in plants treated with Si compared to control. In Si treatments, CAT activity was increased to 12%. Tale Ahmad [53] plants exposed to Si showed a significant increase in the activity of CAT compared to the control. In Si treatment, catalase activity was subsequently increased to 12%. POD plays a vital role in eliminating malondialdehyde resisting cell peroxidation of membrane lipids, reducing the accumulation of hydrogen peroxide, and maintaining cell membrane integrity. By Si application, peroxidase and superoxide dismutase activity were increased to 72.5% and 28.45%, respectively, compared to the control treatment.
